# Validation of a Vaginal Birth after Cesarean Delivery Prediction Model in Teaching Hospitals of Addis Ababa University: A Cross-Sectional Study

**DOI:** 10.1155/2020/1540460

**Published:** 2020-09-18

**Authors:** Eyaya Misgan, Abel Gedefaw, Shiferaw Negash, Anteneh Asefa

**Affiliations:** ^1^Department of Gynecology and Obstetrics, College of Medicine and Health Sciences, Bahir Dar University, Bahir Dar, Ethiopia; ^2^Department of Gynecology and Obstetrics, College of Medicine and Health Sciences, Hawassa University, Hawassa, Ethiopia; ^3^Department of Gynecology and Obstetrics, College of Health Sciences, Addis Ababa University, Addis Ababa, Ethiopia; ^4^School of Public Health, College of Medicine and Health Sciences, Hawassa University, Hawassa, Ethiopia; ^5^Nossal Institute for Global Health, School of Population and Global Health, University of Melbourne, Melbourne, Australia

## Abstract

**Background:**

External validation of a vaginal birth after cesarean delivery (VBAC) prediction model is important before implementation in other settings. The primary aim of this study is to validate the Grobman prenatal VBAC calculator in the Ethiopian setting. Secondarily, the study was aimed at developing and comparing a new VBAC model that includes both the prenatal and intrapartum variables.

**Methods:**

A cross-sectional survey was conducted, complemented by a medical chart review of 268 women admitted at three teaching hospitals of Addis Ababa University and who underwent a trial of labor after one prior cesarean birth. Maternal age, prepregnancy BMI, prior vaginal delivery, prior VBAC, and prior cesarean delivery indication type were included in the Grobman model. Observed delivery outcomes were recorded and then compared with the outcomes predicted by the calculator. We assessed the predictive abilities of the Grobman model and the new model using a receiver operating characteristic (ROC) curve. Multivariate logistic regression analysis was conducted to identify variables associated with successful VBAC.

**Results:**

Out of the 268 participants, 186 (69.4%) (95% CI 57.5-81.3) had successful VBAC. The area under the ROC curve (AUC) of the Grobman model was 0.75 (95% CI 0.69-0.81). Notably, the novel model including both the prenatal and intrapartum variables had a better predictive value than the original model, with an AUC of 0.87 (95% CI 0.81-0.93). Prior VBAC, prepregnancy BMI, fetal membrane status, and fetal station at admission were predictors of VBAC in the newly developed logistic regression model.

**Conclusions:**

The success rate of VBAC was similar to other sub-Saharan African countries. The Grobman model performed adequately in the study setting; however, the model including both the prenatal and intrapartum variables was more predictive. Thus, intrapartum predictors used in the new model should be considered during intrapartum counseling.

## 1. Introduction

The increasing cesarean delivery rate in both the developed and developing countries, including Ethiopia, raises concerns regarding the management of subsequent deliveries after cesarean delivery [1]. In Ethiopia, the national cesarean section rate increased from 0.7% in 2000 to 1.9% in 2016, with increases across all administrative regions. Addis Ababa had the highest cesarean section rate (21.4%) in 2016 and the greatest increase since 2000 [2]. Trial of labor after cesarean delivery (TOLAC) represents one of the major changes in obstetric practice in recent times and has been considered a key method for the reduction of the cesarean delivery rate [3]. The American College of Obstetricians and Gynecologists (ACOG) [4] and the Royal College of Obstetricians and Gynaecologists (RCOG) [5] agree that women with a history of one previous low transverse cesarean delivery, a clinically adequate pelvis, and no prior classical uterine scar or rupture are good candidates to attempt a vaginal birth after cesarean delivery (VBAC), provided that they deliver at an institution staffed by physicians and anesthesiologists with adequate resources.

After a cesarean birth, the mode of delivery in a subsequent pregnancy depends on the presence or absence of any contraindications for TOLAC. Appropriate information about the risks and benefits of TOLAC or repeat elective cesarean delivery are necessary for an informed decision [5–8]. During the counseling process, it is important to provide a woman with information about her chances of success as well as the maternal and neonatal risks and benefits associated with a trial of labor [6–9].

Several VBAC prediction models have been developed to support the counseling process and informed decision-making [10–13]. Some of the models use antepartum variables collected during antenatal visits [10], whereas others use both the antepartum and intrapartum variables to predict the probability of successful TOLAC at admission for labor and delivery service [11–13]. The most utilized and validated model in the United States and Europe is the one first reported by Grobman et al. in 2007 [10]. The model is based on six maternal characteristics—age, body mass index (BMI) (kg/m^2^), race, prior vaginal delivery, prior VBAC, and a recurring indication for cesarean delivery—that can be obtained at the first prenatal visit [10]. The probability of VBAC can be determined by entering these characteristics into a simple calculator [14]. The model was internally validated in an independent cohort of clients [15, 16] and later validated externally in Canada [17], Japan [18], Australia [19], and the Netherlands [20]. The model was found to be similarly valid and useful in predicting VBAC success in these countries as it was in the United States [17–20].

To the best of our knowledge, the Grobman model has not been validated in Africa. The current study was aimed at validating the Grobman prediction model [10] using variables collected at the first prenatal visit. We hypothesized that the prenatal Grobman VBAC prediction model would not apply to the Ethiopian population because the predictors of VBAC success are likely to be different in resource-limited settings. In addition, the study identified additional predictors of VBAC success and developed a modified predictor model including both the antepartum and intrapartum variables.

## 2. Materials and Methods

### 2.1. Study Design and Setting

An institution-based cross-sectional study complemented by a review of participants' medical charts was conducted at three teaching hospitals (Tikur Anbessa Specialized Hospital (TASH), Zewditu Memorial Hospital (ZMH), and Gandhi Memorial Hospital (GMH)) associated with Addis Ababa University between April 2015 and January 2016. The hospitals provide 24-hour obstetrics and gynecology (Ob-Gyn) care and have more than 15,000 annual deliveries. In 2014, the proportion of CS deliveries in TASH, ZMH, and GMH was 36.2%, 35.1%, and 32.3%, respectively. Most of the deliveries and evaluations are performed by Ob-Gyn residents under the supervision of Ob-Gyn faculty from Addis Ababa University. All hospitals offer TOLAC with client consent if the following conditions are fulfilled: (1) the mother has one previous lower uterine segment scar, (2) nonrecurring previous indications, (3) an adequate pelvis as assessed by clinical pelvimetry, (4) a singleton pregnancy, (5) cephalic presentation, (6) estimated fetal weight less than 4 kg, and (7) no other current obstetric indications for cesarean delivery. Maternal candidacy for TOLAC is determined just prior to 36 weeks of gestation. Intermittent auscultation with Pinard fetoscope is the common method of intrapartum fetal monitoring in the study settings.

### 2.2. Study Subjects

The study population included all pregnant women with one previous cesarean delivery scar who consented to TOLAC and were admitted to the labor ward for delivery during the study period. All women who fulfilled the aforementioned conditions for TOLAC were consecutively enrolled in the study. Successful VBAC was defined in this study as vaginal delivery of the fetus (spontaneous or instrument-assisted), regardless of neonatal and maternal complications.

### 2.3. Sampling

The sample size was calculated based on several assumptions. First, at least 10 events were collected for each potential predictor of VBAC that were evaluated in the multivariable regression analysis [20]. An event is defined as the least frequent outcome status: failed VBAC, in the context of this study. Second, since there is no previous study on the VBAC success rate in Ethiopia, we used the sub-Saharan estimated event rate of failed VBAC of 31% (95% CI 25%-37%) [21]. In order to develop a model with 10 potential predictors, at least 100 events are required [22]. Hence, a sample size of at least 270 subjects was required (100/37∗100). Based on this sample size and considering the delivery rate at the hospitals during the pretest period, at least 10 months of data collection were required.

### 2.4. Data Collection, Processing, and Analysis

Primary data were collected through face-to-face interviews with women, using a structured and pretested questionnaire. Secondary data were extracted from participants' medical records. Data were collected by resident physicians after delivery and before discharge from the hospitals. Training for the data collectors, pretesting data collection tools, and close supervision during the data collection period ensured high-quality data.

Data were checked for completeness, coded, and entered into IBM SPSS Statistics for Windows (V 21.0, IBM Digital Analytics, Armonk, NY, USA). Descriptive statistical analyses were performed for both the successful and failed VBAC using proportions expressed as percentages. Chi-squared tests (*χ*^2^) or Fisher's exact tests were used to determine statistically significant differences between categorical variables. Continuous variables were summarized using means and standard deviations.

Five of the six variables included in the Grobman model were collected at the first prenatal visit. These included maternal age, prepregnancy BMI, prior vaginal delivery, prior VBAC, and whether the indication for prior cesarean delivery was arrest of dilation or descent. We did not include race as a variable since there is no considerable racial variation in the population of Ethiopia. Moreover, race was not a significant factor in the final models of a study that included a new simple score to predict the success of VBAC in labor [12] or a recent validation study among a diverse United States population [13]. Prenatal variables were extracted from women's medical charts and entered into a formula that calculated each individual woman's predicted VBAC success rate. The prediction probability was divided into 10 deciles (0-10%, 11-20%, 21-30%, etc.). In each category, the actual proportion of observed success was determined. The predictive capacity of the model was established by calculating the area under the receiver operating characteristic (ROC) curve (AUC). The area under the ROC curve was determined nonparametrically, using the trapezoidal rule. Furthermore, we computed the Hosmer and Lemeshow (H-L) goodness-of-fit statistic as a quantitative measure of accuracy.

We also developed an additional multivariate logistic regression model to predict successful VBAC, which included both antepartum variables (age, parity, prepregnancy BMI, prior vaginal delivery, prior VBAC, and previous cesarean delivery indication) and intrapartum variables (cervical effacement, cervical dilatation, fetal station, and amniotic fluid status at admission) based on reports of previous studies [11, 12, 23, 24]. The assessment of cervical dilatation, effacement, fetal head station, and membrane status is part of intrapartum monitoring and was conducted by Ob-Gyn residents. Cervical dilation was assessed in centimeter (cm) which ranged from closed cervices (0 cm) to fully dilated (10 cm); cervical effacement was recorded as a percentage of effacement (0–100%); and fetal head station was assessed based on the location of the fetal head's lowermost portion in the pelvic canal in relation to the ischial spines. The station above and below the ischial spine were categorized as the high and low stations, respectively. Amniotic membrane status was recorded as rupture or intact during admission.

The multivariate logistic regression models were developed using a backward stepwise elimination method. First, we performed bivariate analyses to identify variables that could be related to successful VBAC. Variables with a *P* value of less than 0.2 in the bivariate analysis were included in the multivariate logistic regression analysis. Odds ratios with 95% confidence intervals (CI) were computed to identify and evaluate the strength of VBAC predictors. *P* values less than 0.05 indicated statistical significance. To determine predictive capacity, we constructed a logistic regression model with the model variables, and the AUC was subsequently calculated.

## 3. Results

### 3.1. Sociodemographic Characteristics of the Study Participants

During the ten-month study period, the total number of deliveries in the hospitals was 12,916, including 4,520 (35%) deliveries by cesarean section. Only 497 (3.9%) women who delivered during this period had a history of one previous cesarean delivery. Of these, 129 (65%) were candidates for TOLAC but indicated a preference for repeat CS during admission. The remaining 86 (35%) were not candidates for TOLAC and underwent repeat CS, leaving 282 women who fulfilled the inclusion criteria. Of those who met the criteria, 14 (5%) were excluded due to lack of consent or incomplete data. The final analyses included 268 participants.

Table 1 describes sociodemographic characteristics of study participants. The mean prepregnancy body mass index (BMI) of the participants was 25.8 kg/m^2^ (±4.6). There was a significant difference in the mean BMI of participants with successful (24.5 ± 3.6) and failed VBAC (28.7 ± 5.4) (*P* < 0.001). Age, marital status, occupation, and religion were not significantly associated with successful or failed VBAC.

### 3.2. Obstetric Characteristics of the Study Participants

Table 2 describes the current and past obstetric characteristics of study participants. One hundred fifty-seven (58.6%) participants had a history of only one cesarean delivery and were admitted for the first TOLAC. Among these participants, 60.5% (95/157) had successful VBAC and 39.5% (62/157) had failed VBAC. The remaining 111 (41.4%) participants had given birth two or more times before the current pregnancy, either by cesarean or by vaginal delivery. During admission to the labor ward for TOLAC, 118 (44%) participants had cervical dilation of at least 5 cm and the amniotic membrane was ruptured spontaneously for 121 (45%) of the participants.

### 3.3. Success Rate of VBAC and Its Predictors

Table 3 describes the logistic regression analysis of factors associated with VBAC using the antepartum and intrapartum variables. Out of 268 women who participated in the study, 186 (69.4%) (95% CI 57.5-81.3) had successful VBAC. In the bivariate logistic regression, parity, previous vaginal delivery, previous VBAC, prepregnancy BMI, amniotic membrane status, fetal station, and cervical effacement at admission significantly predicted VBAC success at *P* < 0.2. However, in the final multivariate regression model, only prior VBAC, prepregnancy BMI, membrane status, and fetal station at admission had a statistically significant association with VBAC success (*P* < 0.05).

Women who had prior VBAC history were 16 times more likely to have a repeat VBAC than those who had not had a prior VBAC (aOR 16.74; 95% CI 3.99-70.19). The odds of successful VBAC for women with normal prepregnancy BMI (BMI < 25 kg/m^2^) was twelve times higher than those who were overweight or obese (BMI ≥ 25 kg/m^2^) (aOR 11.87; 95% CI 15.46-28.34). Women who had spontaneous ruptured membranes at admission were almost three times more likely to have successful VBAC compared to women with intact membranes at presentation (aOR 2.67; 95% CI 1.28-5.57). Finally, the odds of having a successful VBAC was 90% lower for women with a high station (above 0 station on pelvic examination) at admission (aOR 0.10; 95% CI 0.04-0.25).

### 3.4. Validation of the Prediction Model

#### 3.4.1. Distribution of Probabilities of the Grobman and Newly Developed Models

Table 4 displays predictions according to the Grobman VBAC model. In this population, the Grobman model predicted a score above 60% for 255 (95.1%) participants and above 80% for 158 (58.9%) participants. Thirteen participants (4.8%) had a predicted score below 60%. The median (IQR) predicted score was 81.5% (74.9-93.9), with a minimum predicted score of 45.5% and a maximum prediction of 97.5%.

The newly developed model, which incorporates both the prenatal and intrapartum factors, resulted in significantly higher predicted probabilities for those who ultimately had a successful VBAC, compared to those who had repeat emergency cesarean deliveries (median (IQR) = 83.8% (78.4-94.8) and 74.8% (70.7-82.1), respectively, *P* < .001).

#### 3.4.2. Discriminative Performance of the Grobman and Newly Developed Models

Discriminative performance of the Grobman prediction model is shown in Figure 1. The area under the ROC curve (AUC) was 0.75 with 95% CI (0.69-0.81) and *P* < 0.001, indicating good discriminative ability. The goodness of calibration was supported by a nonsignificant H-L statistic (*P* < 0.262). For a predicted score of 80%, the sensitivity and specificity of the model to predict the chance of success were 97.3% and 90.2%, respectively. In contrast, for a predicted score of 60%, the sensitivity and specificity of the model in predicting success were 71.0% and 31.7%, respectively.

Figure 1(b) shows discriminative performance of the newly developed model including the prenatal and intrapartum variables. This model had a mean predictive probability of successful VBAC of 69.4% (±30.1). Only 27% of the participants had predicted probabilities below 60%. The median (IQR) predictive chance was 81% (45.5-95.9). The ROC of our model has an AUC of 0.87 (95% CI 0.81-0.93), which indicates a good discriminative ability.

## 4. Discussion

VBAC has long been proposed as a viable measure to reduce overall cesarean delivery rates in both the low- and middle-income and high-income countries [4–6]. A study conducted in sub-Saharan Africa reported that VBAC is safe and its success rates range between 60% and 80% if complemented with careful client selection and good management of labor [21]. However, important challenges related to VBAC trialing exist in low-income settings like Ethiopia, where there are bottlenecks in the ability to provide high-quality intrapartum care, including inconsistent availability of comprehensive emergency obstetric care signal functions [25]. In this study, we found that 282/497 (56.7%) women with one previous CS delivery had TOLAC. This finding is consistent with the meta-analysis of the sub-Saharan Africa studies that showed a TOLAC rate of 37% to 97% [21]. Moreover, a recent study in Ethiopia also showed the TOLAC rate of 38.5% [26].

In our study, more than two-thirds (69.4%) of the participants had successful VBAC. This finding is similar to the results of a meta-analysis that reported a VBAC success rate of 69% in sub-Saharan African countries [21]. Similarly, other studies also reported comparable levels of VBAC success rates in the United States (71%) [13], India (73%) [25], Ghana (61%) [27], Nigeria (73%) [28], and Egypt (77%) [29]. Some studies also report lower VBAC success rates in Ethiopia (44.5%) [26], Nigeria (45.1%) [30], and Brazil (45%) [31]. The VBAC success rate in the present study was lower than that in the studies in Japan (91.5%) [18], Australia (83%) [19], and China (80%) [32], which might be due to variation in the maternity care system between Ethiopia and these countries.

The variation in VBAC success rates among different studies could be due to different criteria for TOLAC and differences in predictors of VBAC [33], such as past obstetric performance like prior VBAC, ethnic differences, prior vaginal delivery, and indication for prior cesarean delivery. The relatively high rate of the successful VBAC revealed in the present study might also reflect the meticulous selection of cases for the provision of TOLAC, as the health centers where the study took place are tertiary and teaching hospitals for the undergraduate and postgraduate students. This high degree of cumulative probability of VBAC success should be used to counsel pregnant women for the subsequent mode of delivery in similar settings.

Prior to this study, there was no locally validated VBAC prediction model to counsel Ethiopian women on decisions about the mode of delivery. Without population-validated and evidence-based calculators for successful TOLAC, women are counseled based on physicians' experiences and evidence from other countries, which could lead to biased decisions, as has been demonstrated in high-income countries [34]. These biases may have negatively impacted acceptance of TOLAC among eligible women in the study hospitals. Validation of a predictive model could provide tailored information by estimating the risk of emergency cesarean delivery in a specific context. Moreover, an evidence-based counseling process could be standardized among many health care providers in a given setting.

The Grobman prenatal VBAC prediction allows the determination of a patient-specific chance for successful VBAC using six variables that can be ascertained at the first prenatal visit [10]. There were attempts to develop VBAC predictor models before the Grobman model; however, these were not widely applicable for use in clinical practice [35–38]. One of the main reasons why these models, including the Flamm score, failed was the inclusion of intrapartum variables [35]. The Flamm VBAC predictor scoring was developed and tested using five variables that are assessed at hospital admission for labor [35]. Therefore, unlike the Grobman model, the Flamm scoring system would not be valid for use before the onset of labor where evidence for counseling is critical. However, the Flamm score is important for women who initially opt for trial of labor but later change their mind after the onset of labor [35]. Additionally, the Flamm score has been used to refine other prediction models, including the Grobman model [10]. Cognizant of the importance of intrapartum variables to predict VBAC precisely, Grobman et al. developed a modified prediction model in 2009 that includes both the antepartum and intrapartum variables [11].

In this study, we chose to validate the Grobman prenatal VBAC prediction model [10] in our setting instead of the intrapartum prediction model [11]. The prenatal prediction model showed greater clinical advantage than the intrapartum prediction model for the reduction of repeat CS and can be used for counseling and decision-making about TOLAC during the antenatal period and before the onset of labor [10]. The prenatal prediction model variables are also less likely to be affected by interobserver variability, particularly in low-resource settings, where intrapartum variables like cervical dilatation and effacement are often affected by the quality of health care and experience of health care providers [39]. The validated prediction model can be used across the spectrum of health care settings.

This study confirms that the prenatal Grobman VBAC success prediction model is applicable in the Ethiopian context with similar efficacy to that observed in the USA. The AUC of the validated model in our context (0.75, 95% CI 0.69-0.81) is the same as that of the original model (0.75, 95% CI 0.74-0.77) [10]; the slightly wider confidence interval of the validated model in our context could be due to the small sample size of our study. Our validation showed better fitness as compared to the external validations in the USA with two independent cohorts of patients (AUC = 0.72; 95% CI 0.65-0.74 [15] and AUC = 0.70; 95% CI 0.65-0.74 [16]), as well as external validations in Canada (AUC = 0.72; 95% CI 0.70-0.74) [17], the Netherlands (AUC = 0.68; 95% CI 0.63-0.72) [20], and Australia (AUC = 0.71; 95% CI 0.67-0.76) [19]. However, the AUC in our study was slightly lower compared to that in the Japanese cohort where the AUC was 0.81 (95% CI 0.75-0.87) [18].

Despite the good performance of the validated Grobman prenatal VBAC prediction model in our setting, we found that the new, locally developed model using both the prenatal and intrapartum variables had better predictive performance, with an AUC of 0.87 (95% CI 0.81-0.93). The performance of the locally developed model was also better than that of the Grobman prediction model including intrapartum variables, with an AUC of 0.77 (95% CI 0.76-0.78) [11]. The wide confidence interval in our study is likely due to the small size of the participants. Our new VBAC prediction model also supported the theory that data available at admission can improve prediction of a successful VBAC [11].

This is the first validation of a VBAC prediction model in the Ethiopian setting. In comparison to other validation studies, the performance of the prediction model in our study population is good. However, when making a decision about the mode of delivery after previous cesarean delivery, we consider it helpful to distinguish between women with a high or low probability of VBAC and those with a moderate probability. This will help pregnant women with a prior cesarean delivery make an informed decision about a TOLAC or a planned cesarean delivery. Although our dataset was smaller than those of other studies, we achieved an adequate sample size for testing and developing a model. Because it includes both the antepartum and intrapartum predictors based on previous studies of VBAC prediction [11, 12, 23, 24], it is likely that the new prediction model will provide a more appropriate and applicable alternative for our study population than the existing models.

As this study was conducted in tertiary hospitals, the findings are not necessarily generalizable to other settings where VBAC occurs. Additionally, our study setting may differ from other settings in terms of intrapartum fetal monitoring, the threshold level for TOLAC, client volume, and quality of health care services, making comparisons difficult across regions or countries. Further validation studies involving lower-level hospitals like the general and primary hospitals in Ethiopia are warranted. However, despite differences in setting, the validated Grobman VBAC calculator and the newly identified intrapartum VBAC predictor variables may improve the process of informed decision-making for women and health care providers during antepartum and intrapartum care.

Incomplete data for a few participants also limited this study to some extent. Prepregnancy weight and previous indication for cesarean delivery were missing from some participants' medical chart. Additionally, some women had their previous cesarean deliveries in birth centers that were not involved in this study. For those women, perceived weight and indication for cesarean delivery were based on client recall, which can be prone to recall bias. However, the number of missing observations were relatively few (three for prepregnancy weight and four for the previous indication for cesarean section) and thus do not significantly affect the results of the validation test.

## 5. Conclusion

The success rate of VBAC was found to be similar to other sub-Saharan African countries. Hence, VBAC remains a viable option for clients with one prior cesarean delivery in our study setting. Additionally, external validation of the predictive model developed by Grobman and colleagues performed adequately in our setting. Therefore, the model may be used in practice to refine the antepartum counseling process. However, the intrapartum predictors identified by this study should be considered in decision-making processes when women present during the intrapartum period.

## Figures and Tables

**Figure 1:** (a) Receiver operating characteristic (ROC) curve for the Grobman VBAC prediction model. (b) Receiver operating characteristic (ROC) curve of the newly developed VBAC prediction model.

**Table 1:** Sociodemographic characteristics of study participants (*n* = 268).

Variables	Successful VBAC; 186 (69.4%)	Failed VBAC; 82 (30.6%)	*P* value
	Number (%)	Number (%)	
Age in years (mean ± SD)	29 ± 3.7	28 ± 4.3	0.05
20-24	19 (10.2)	16 (19.5)	0.194
25-29	93 (50)	38 (46.3)	
30-34	52 (28.0)	18 (22.0)	
≥35	22 (11.8)	10 (12.2)	
Religion			0.046
Orthodox Christian	120 (64.5)	40 (48.8)	
Muslim	41 (22.0)	24 (29.3)	
Protestant	25 (13.4)	18 (22.0)	
Marital status			0.906
Married	181 (97.3)	80 (97.6)	
Others^∗^	5 (2.7)	2 (2.4)	
Educational status			0.018
Above secondary	19 (10.2)	8 (9.8)	
Secondary (9-12)	90 (48.4)	28 (34.1)	
Primary (1-8)	63 (33.9)	30 (36.6)	
No formal education	14 (7.5)	16 (19.5)	
Occupation			0.168
Currently working	51 (27.4)	16 (19.5)	
Housewife	135 (72.6)	66 (80.5)	
Prepregnancy BMI (mean ± SD)	24.5 ± 3.6	28.7 ± 5.4	<0.0001
<25	112 (60.2)	18 (22.0)	<0.001
≥25	74 (39.8)	64 (78.0)	

^∗^Divorced, widow, and single. BMI: body mass index.

**Table 2:** Past and current obstetric performance of study participants (*n* = 268).

Variables	Successful VBAC; 186 (60.4)	Failed VBAC; 82 (30.6%)	*P* value
	Number (%)	Number (%)	
Parity			<0.001
Primiparous (para 1)	95 (51.1)	62 (75.6)	
Multiparous (≥2)	91 (48.9)	20 (24.4)	
Prior vaginal delivery			<0.001
Yes	91 (48.9)	18 (22)	
No	95 (51.1)	64 (78)	
Prior VBAC			<0.001
Yes	71 (38.2)	4 (4.9)	
No	115 (61.8)	78 (95.1)	
Prior cesarean delivery indication			0.303
Recurring	23 (12.4)	14 (17.1)	
Nonrecurring	163 (87.6)	68 (82.9)	
Place of antenatal care			<0.001
Health center	115 (61.8)	70 (85.4)	
Hospital	71 (38.2)	12 (14.6)	
Antenatal care initiation time			<0.001
1st trimester	87 (46.8)	70 (85.4)	
2nd trimester and above	99 (53.2)	12 (14.6)	
Fetal gestational age			0.529
37-39^6/7^ weeks	103 (55.4)	42 (51.2)	
40-41^6/7^ weeks	83 (44.6)	40 (48.8)	
Cervical dilatation			0.298
<5 cm	108 (58.1)	42 (51.2)	
≥5 cm	78 (41.9)	40 (48.8)	
Cervical effacement			0.004
<50%	20 (10.8)	20 (24.4)	
≥50%	166 (89.2)	62 (75.6)	
Fetal station			<0.001
High (<0)	101 (54.3)	72 (87.8)	
Low (≥0)	85 (45.7)	10 (12.2)	
Fetal amniotic membrane			0.063
Ruptured	77 (41.4)	44 (53.7)	
Intact	109 (58.6)	38 (46.3)	

**Table 3:** Logistic regression analysis of factors associated with VBAC using the antepartum and intrapartum variables.

Variables	VBAC		COR (95% CI)	*P* value	aOR (95% CI)	*P* value
	Yes	No				
Parity				0.012		0.466
Primiparous	95	62	0.38 (0.17-0.81)		2.94 (0.16-53.4)	
Multiparous	91	20	1		1	
Prior vaginal delivery				0.006		0.357
Yes	91	18	3.02 (1.37-6.63)		4.05 (0.21-79.47)	
No	95	64	1		1	
Prior VBAC				0.001		≤0.001
Yes	71	4	12.29 (2.83-53.18)		16.74 (3.99-70.19)	
No	115	78	1		1	
Prepregnancy BMI				≤0.001		≤0.001
<25	112	18	5.38 (2.95-9.80)		11.87 (15.46-28.34)	
≥25	74	64	1		1	
Membrane status				0.064		0.009
Ruptured	77	44	1.64 (0.97-2.77)		2.67 (1.28-5.57)	
Intact	109	38	1		1	
Cervical effacement				0.044		0.360
<50%	20	20	0.40 (0.17-0.97)		0.64 (0.25-1.66)	
≥50%	166	62	1		1	
Fetal station				≤0.001		≤0.001
High (<0)	101	72	0.16 (0.06-0.42)		0.10 (0.04-0.25)	
Low (≥0)	85	10	1		1	

COR: crude odds ratio; aOR: adjusted odds ratio; BMI: body mass index.

**Table 4:** Grobman VBAC prediction model outcomes of the predicted compared with the observed VBAC success rate.

Decile group	Number predicted	Number observed	Observed VBAC (%)
0-10	0	0	n/a
10-20	0	0	n/a
20-30	0	0	n/a
30-40	0	0	n/a
40-50	5	3	60
50-60	8	2	25
60-70	25	13	52
70-80	72	36	50
80-90	72	50	69.4
90-100	86	82	95.3

n/a = not applicable.

## Data Availability

All available data and materials are included in the manuscript.

## Abbreviations

aOR: Adjusted odds ratio
AUC: Area under the ROC curve
BMI: Body mass index
CI: Confidence interval
ROC: Receiver operating characteristic
TOLAC: Trial of labor after cesarean delivery
VBAC: Vaginal birth after cesarean delivery.
